The article "Clinical Observation of the Effect of Nasal Breathing on Nonanalgesic and Sedative Gastroscopy" was retracted in 2023. Reasons: signs of a paper mill; suspected computer-generated content; unreliable results or conclusions; concerns about the data.

# Clinical Observation of the Effect of Nasal Breathing on Nonanalgesic and Sedative Gastroscopy

**DOI:** 10.1155/2022/8603625

**Published:** 2022-08-26

**Authors:** Xuzhen Zhang

**Affiliations:** Digestive Endoscopy Center, Beijing Jingmei Group General Hospital, Mentougou, Beijing 102399, China

## Abstract

This study aimed to investigate the safety, tolerance, and comfort of the subjects in gastroscopy by observing and comparing the effect of gastroscopy under two different breathing modes: nasal breathing and nasal inspiration and oral expiration. A total of 60 subjects who underwent routine gastroscopy in the hospital from January 2021 to June 2021 were selected as the research subjects. According to the willingness of the subjects, they were divided into a nasal breathing group and a nasal inspiration and oral expiration group. The differences in vital signs, adverse reactions, and visual analog scale (VAS) scores were compared between the two groups. There were no significant differences in mean arterial pressure, heart rate, and blood oxygen saturation between the two groups before, during, and after the examination (*P* > 0.05). The nasal breathing group had fewer adverse reactions such as nausea, cough, belching, and restlessness than the nasal inspiration and oral expiration group, and the difference was statistically significant (*P* < 0.01). VAS score of the nasal breathing group was lower than that of the nasal inspiration and oral expiration group, and the difference was statistically significant (*P* < 0.01). Subjects are more tolerant to nasal breathing mode, which causes fewer adverse reactions, less pain, and more comfort and is more worthy to be popularized in primary hospitals.

## 1. Introduction

Due to its intuitive and clear features, gastroscopy is widely used in clinical practice and is a common method for the diagnosis and treatment of gastrointestinal diseases [1, 2]. Although more and more sedative and analgesic gastroscopes are currently being carried out, the technical requirements for anesthesiologists and the higher cost of gastroscopy compared with nonanalgesic and sedative gastroscopy limited its widespread development in primary hospitals [3]. The application of sedatives and analgesics can effectively narrow the discomfort during gastroscopy. However, the inhibitory effect of narcotic drugs on the cardiovascular system can result in hypotension and even coma. Some subjects have adverse reactions such as nausea and vomiting after examination. Some scholars have found that many subjects did not choose sedative and analgesic gastroscopy for fear of adverse reactions related to anesthesia [4], so there is still a high objective demand for nonanalgesic and sedative gastroscopy in the examined population. This study observed and compared the application effects of nasal breathing and nasal inspiration and oral expiration in nonanalgesic sedative gastroscopy and discussed the safety, tolerance, and comfort of the two breathing methods.

The article "Clinical Observation of the Effect of Nasal Breathing on Nonanalgesic and Sedative Gastroscopy" was retracted in 2023. Reasons: signs of a paper mill; suspected computer-generated content; unreliable results or conclusions; concerns about the data.

## 2. Materials and Methods

### 2.1. General Information

This prospective cohort study was performed at the Digestive Endoscopy Center, Beijing Jingmei Group General Hospital. The study was endorsed by the Ethics Committee of Beijing Jingmei Group General Hospital (no. 2020KY018-01), and informed consent was obtained from all patients. A total of 60 subjects who underwent nonanalgesic and sedative gastroscopy in the Digestive Endoscopy Center of Beijing Jingmei Group General Hospital from January 2021 to June 2021 were selected as the research subjects. The subjects were divided into 2 groups according to their wishes: the nasal breathing group (group A, *n* = 30) and the nasal inhalation and oral expiration group (group B, *n* = 30). There were 28 males and 32 females, aged 18 to 78 years, with an average of 50.87 years, and body mass index (BMI) of 17.69 to 32.46. The *P* values of the two groups in terms of age and BMI were all greater than 0.05, and the difference was not statistically significant (see Table 1). The inclusion criteria were as follows: (1) those with smooth nasal breathing; (2) those with no contraindications for gastroscopy; and (3) those with informed consent and who voluntary participated in the study. The exclusion criteria were (1) those with nasopharynx or oropharyngeal airway obstruction; (2) those who had contraindications to gastroscopy, such as serious cardiovascular diseases accompanied by cardiac insufficiency or serious coronary heart disease, descending aortic aneurysm, serious lung diseases, serious oral or throat diseases, endoscopy failure, acute tonsillitis, acute pharyngitis, corrosive esophagitis, suspected gastrointestinal perforation, and extreme systemic failure; (3) those who refused endoscopy; (4) those who were mentally abnormal and unable to cooperate; (5) those who proposed transnasal gastroscopy; and (6) those who proposed sedative and analgesic gastroscopy [5].

### 2.2. Research Methods

#### 2.2.1. Routine Preparations

The subjects were explained about the purpose of the examination, the matters that need cooperation, and the related risks and complications that might occur during and after the examination. They signed the informed consent. All subjects were forbidden to eat or drink for more than 8 hours before the examination.

#### 2.2.2. Operation Method

The subjects were given 10 ml of dyclonine hydrochloride mucilage (Yangtze River Pharmaceutical Co. Ltd., 10 ml: 0.1 g) 10 minutes before gastroscopy, to anesthetize the throat and oral cavity for 3 to 5 minutes, which they eventually swallowed. After that, they were placed in the left lateral decubitus position and connected with the multifunctional monitor. Subjects in group A adopted nasal breathing mode during the whole process of gastroscopy (see Figure 1), and which was performed after their breathing was stable. Subjects in group B adopted the mode of nasal inspiration and oral expiration throughout the examination (see Figure 2), and the rest were the same as that in group A.

The article "Clinical Observation of the Effect of Nasal Breathing on Nonanalgesic and Sedative Gastroscopy" was retracted in 2023. Reasons: signs of a paper mill; suspected computer-generated content; unreliable results or conclusions; concerns about the data.

### 2.3. Observation Indicators

The mean arterial pressure (MAP), heart rate (HR), and blood oxygen saturation (SpO2) changes of the two groups of subjects were monitored and recorded before the start of the examination, during the operation (that is, when the endoscope passes through the gastroesophageal junction), and after the end of the examination. The adverse reactions of the two groups during gastroscopy, including nausea, cough, belching, and restlessness, were observed and recorded. The subjects were given a visual analog scale (VAS) score immediately after the gastroscopy that reflected the subject's personal feelings [6] (method: use a 10 cm ruler as a scale plate: “0” means no pain, “10” indicates extremely severe pain; the higher the score, the more severe the pain). The differences in VAS scores between the two groups were accounted for and compared (see Figure 3).

### 2.4. Statistical Analysis

SPSS 26 software was used for statistical analysis. Quantitative data were expressed as mean ± standard deviation ($\bar{x}\pm s$), and analyzed by t-test. Qualitative data Were expressed as use cases (%) and analyzed by Chi-square test. P < 0.05 was considered statistically significant.*P* < 0.05 was considered statistically significant.

## 3. Results

### 3.1. Comparison of Vital Signs between the Two Groups of Subjects before, during, and after Examination

Before examination, HR, MAP, and SpO2 values of the two groups were not statistically significant (*P* > 0.05). During the examination, that is, when the endoscope passed through the gastroesophageal junction, the MAP and HR values of the two groups were increased, and the difference between the two groups was not statistically significant (*P* > 0.05). There was no meaningful change in SpO2 between the two groups, and the difference was not statistically significant (*P* > 0.05). After the examination, the MAP and HR of subjects basically recovered to the levels before the examination, and there was no noteworthy change in SPO2, and the difference was not statistically significant (*P* > 0.05). See Table 2.

The article "Clinical Observation of the Effect of Nasal Breathing on Nonanalgesic and Sedative Gastroscopy" was retracted in 2023. Reasons: signs of a paper mill; suspected computer-generated content; unreliable results or conclusions; concerns about the data.

### 3.2. Comparison of the Inspection Completion Rate of the Subjects in the Two Groups

The inspection completion rate of the subjects in group A was 100%, which was higher than that in group B (96.67%); however the difference was not statistically significant (*P* > 0.05, see Table 3).

### 3.3. Comparison of Adverse Reactions in the Examination of the Two Groups of Subjects

The two groups of subjects had different degrees of adverse reactions during the examination, mainly belching, nausea, cough, and throat discomfort. The adverse reactions of the subjects in group A were significantly less than those in group B, and the difference was statistically significant between the two groups (*P* < 0.01, see Figure 4). Among various adverse reactions, the incidence of nausea in group A was lower than that in group B, and the difference was statistically significant (*P* < 0.05, see Table 4), while for other adverse reactions such as belching, cough, throat discomfort, restlessness, and suffocation, there was no significant difference between the two groups (*P* > 0.05, see Table 4).

### 3.4. Comparison of VAS Scores between the Two Groups of Subjects

Comparison between the two groups showed that the VAS score of group A was less than that of group B, and the difference between group A and group B was statistically significant (*P* < 0.01, see Figure 5).

## 4. Discussion

Due to its low cost, nonanalgesic and sedative gastroscopy can be carried out in primary hospitals without the limitations related to the technical level of anesthesiologists and anesthetic drugs, and it still has certain objective needs. At present, more and more analgesic and sedative gastroscopy is carried out, but there are also some patients who choose nonanalgesic and sedative gastroscopy when they re-examine after experiencing analgesic and sedative gastroscopy, because they are worried about the re-occurrence of adverse reactions of anesthesia-related gastroscopy. However, the adverse reactions associated with nonanalgesic sedation gastroscopy and its low comfort have been the main reasons for improving patient compliance. Therefore, reducing the subject's rejection and fear of nonanalgesic and sedative gastroscopy and the discomfort during the examination process has become the inevitable problem and the focus of attention of the current digestive endoscopists. Liao et al. found that the inspection effect of magnetic control capsule endoscopy is comparable to that of traditional gastroscope, and the subjects have better tolerance [7]. Chen et al. found that acupuncture can reduce the adverse reactions related to gastroscopy [8], and this study found that nasal breathing can reduce the incidence of nonanalgesic and sedative gastroscopy-related adverse reactions.

The article "Clinical Observation of the Effect of Nasal Breathing on Nonanalgesic and Sedative Gastroscopy" was retracted in 2023. Reasons: signs of a paper mill; suspected computer-generated content; unreliable results or conclusions; concerns about the data.

Airway ventilation is critical to the subject to maintain a stable life state during nonanalgesic and sedative gastroscopy and is mainly completed by the subject's respiration. During the operation of gastroscopy, the subject adjusts the breathing mode to cooperate with the inspection operation, and the most commonly used breathing modes of the subjects are the nasal inhalation and nasal expiration, namely, the nasal breathing mode and the nasal inspiration and oral expiration mode. The subjects in the nasal breathing group adopted the breathing mode of nasal inhalation and nasal exhalation throughout the operation. In the nasal inspiration stage, the airflow mainly passed through the middle and lower parts of the nasopharynx to the oropharynx, and most of the airflow passed through the front side of the pharynx. It flows into the larynx to complete the inhalation of external gas. During expiration, the airflow mainly passes through the posterior wall of the laryngopharynx to the oropharynx and then flows into the nasal cavity through the posterior wall of the nasopharynx to complete the exhalation of the gas in the body. The subjects in the nasal inspiration and oral expiration group adopted the breathing mode of nasal inspiration and oral expiration throughout the operation process. In this breathing mode, in the nasal inspiration stage, the airflow mainly passed through the middle and lower parts of the nasopharynx to the oropharynx, and most of the airflow passed through the pharynx. In the expiration stage, under the control of nerve, the outlet of the nasal cavity airway is closed and the gas passes through the glossopharyngeal plane and is exhaled from the oral airway, thereby completing the internal and external gas exchange, sustaining a stable blood oxygen saturation, and maintaining a stable state of life.

By observing the application effect of the two breathing modes in nonanalgesic and sedative gastroscopy, this study found that the incidence of nausea, cough, belching, restlessness, and other adverse reactions in the nasal breathing group during gastroscopy was significantly less than that in the nasal inspiration and oral expiration group. By comparing the different adverse reactions of the two groups, it was found that the occurrence of one of the adverse reactions, nausea, in the nasal breathing group was less than that in the nasal inspiration and oral expiration group. There were no significant differences in the occurrence of adverse reactions such as cough, belching, throat discomfort, restlessness, and chest tightness between the two groups. The results of the study showed that the subjects who used the nasal breathing mode to breathe during nonanalgesic and sedative gastroscopy had fewer adverse reactions than the nasal inspiration and oral expiration mode. Especially the incidence rate of nausea in the nasal breathing group was less than that in the nasal inspiration and oral expiration group. The results of this study are not consistent with the results reported by Yang et al. [9]. The main reason for the analysis is that gastroscopy as an invasive operation can cause physical stress in some subjects. When the gastroscope enters the esophagus and stomach cavity through the throat, the physical stimulation to the inner wall causes pharyngeal tension reflex, which leads to the occurrence of adverse reactions such as nausea [10]. For the subjects adopting the nasal inspiration and oral expiration mode, in the expiration stage, the nasal cavity airway outlet is closed under the action of nerve control, and the gas is exhaled from the oral airway after passing through the glossopharyngeal plane. Compared with exhaling through the nose, the maximum flow rate of exhaled gas is increased, and the pressure drop is mainly concentrated in the oral cavity, which doubles during exhalation, resulting in disturbance of the airflow in the laryngeal cavity [11]. When the air flows through the throat and mouth to exhale out of the body, the airflow disorder state and the influence state caused by the gastroscope stimulation overlap, which increases the occurrence and degree of adverse reactions. For the subject adopting the breathing mode of nasal breathing, in the expiration stage, the airflow mainly reaches the oropharynx through the posterior wall of the laryngopharynx and then flows into the nasal cavity through the posterior wall of the nasopharynx, and finally the air is exhaled through the nasal cavity. This process reduces the impact of airflow disturbance in the laryngeal cavity compared with the nasal inspiration and oral expiration mode and also decreases the occurrence of related adverse reactions and the degree of adverse reactions. Therefore, in nonanalgesic and sedative gastroscopy, in subjects adopting the breathing mode of nasal breathing, compared with the nasal inspiration and oral expiration mode, the occurrence of adverse reactions such as nausea, coughing, and belching can be reduced to a certain extent. It can also improve the patient's tolerance to nonanalgesic and sedative gastroscopy to a certain extent.

The article "Clinical Observation of the Effect of Nasal Breathing on Nonanalgesic and Sedative Gastroscopy" was retracted in 2023. Reasons: signs of a paper mill; suspected computer-generated content; unreliable results or conclusions; concerns about the data.

The results of the study showed that the VAS score of the nasal breathing group was significantly lower than that of the nasal inspiration and oral expiration group, indicating that the subjects who adopted the nasal breathing mode during nonanalgesic and sedative gastroscopy were more comfortable than those in the nasal inspiration and oral expiration mode. The main reason for the analysis is that for the subject adopting the breathing mode of nasal inspiration and oral expiration during the nonanalgesic and sedative gastroscopy process, in the expiration stage, the air is often exhaled through the mouth with symptoms such as dry mouth and thirst. These symptoms can lead to sympathetic nerve excitation, which aggravates anxiety and irritability [12]. During nonanalgesic and sedative gastroscopy, the subjects adopted the breathing mode of nasal breathing, which could prevent the exhaled gas from flowing through the glossopharyngeal plane and oral airway, thereby avoiding related symptoms such as dry mouth and thirst. Sympathetic nerve stimulation and excitation [13]can also be avoided, in order to reduce the subject's anxiety and irritability during nonanalgesic and sedated gastroscopy to a certain extent. Therefore, in non-analgesic and sedative gastroscopy, subjects using the breathing mode of nasal breathing, compared with the breathing mode of nasal inspiration and oral expiration, have less discomfort symptoms, feel less pain, and have better tolerance.

In this study, it was found that all the subjects in the nasal breathing group that used the breathing mode of nasal inhalation and nasal exhalation had completed the examination, while in the nasal inspiration and oral expiration group, there was one subject who interrupted the examination and failed to complete the whole process. The results of the study showed that the examination completion rate of the nasal breathing group was greater than that of the nasal inspiration and oral expiration group; however, the difference between the two groups was not statistically significant. The reason may be that for subjects adopting the nasal inspiration and oral expiration mode, in the expiration stage, the airflow in the larynx caused by the exhalation is disordered, which aggravates the discomfort of the subject, and thus makes the subject unable to tolerate and continue to complete the examination, thereby terminating the inspection. The reason may also be related to the individual differences of the subjects. The subjects may have poor tolerance for nonanalgesic and sedative gastroscopy, resulting in their inability to tolerate and cooperate to completing the examination. The exact cause remains to be further confirmed by large sample studies.

Through the study, it was found that the mean arterial pressure and heart rate value of the two groups of subjects increased significantly when the gastroscope passed through the gastroesophageal junction. The two values gradually return to the state before the examination in the end, indicating that the effects of nasal breathing mode and nasal inspiration and oral expiration mode on the subject's hemodynamics are basically the same. After the examination, the subject's hemodynamics can be restored to the state before the examination. The blood oxygen saturation values of the two groups of subjects did not show significant changes in the whole process, indicating that the subjects who underwent nonanalgesic and sedative gastroscopy under the two breathing modes had the same effect on airway ventilation. By comparing the above data, it is found that in nonanalgesic and sedative gastroscopy, subjects can safely cooperate with medical workers to complete the inspection operation whether they use the nasal breathing mode or the nasal inspiration and oral expiration mode. Both breathing modes are safe during the examination. The results of the study also showed that there were no significant differences in mean arterial pressure, heart rate, and blood oxygen saturation between the two groups of subjects before and after nonanalgesic sedation gastroscopy, and no serious complications occurred in any subject, and no case of death occurred. The results of this study showed that there was no difference between the two groups regarding the safety of subjects before and after nonanalgesic sedation gastroscopy. The study also showed that, no matter whether the subjects adopt the nasal breathing mode or the nasal inspiration and oral expiration mode, it will not seriously affect their life safety, and the subjects can maintain a safe state before and after the examination.

The article "Clinical Observation of the Effect of Nasal Breathing on Nonanalgesic and Sedative Gastroscopy" was retracted in 2023. Reasons: signs of a paper mill; suspected computer-generated content; unreliable results or conclusions; concerns about the data.

In order to avoid the influence of different physicians' operations on the research results, all nonanalgesic and sedative gastroscopy procedures involved in this study were performed and completed by the same experienced endoscopist [14]. The operating physician fully communicated with the patient before the examination, explained the purpose of the examination and the precautions that require the cooperation of the subject, and acted gently during the operation, especially when entering the entrance of the esophagus along the posterior pharyngeal wall. If there is resistance, do not blindly and forcefully insert the endoscope; the subject can be asked to swallow, and at the same time, the endoscope can be inserted into the esophagus, so as to prevent damage or tear of the pharyngeal mucosa. The gentle operation of the endoscopist avoided the discomfort and adverse reactions associated with rough operation and also the occurrence of serious complications. The subjects adopted the nasal breathing mode during the nonanalgesic and sedative gastroscopy, which reduced the occurrence of side effects to a certain extent and the pain of the examination; improved the tolerance, comfort, and compliance of the subjects; and thus avoided the delay of the patients' condition caused by the fear of gastroscopy [15].

In conclusion, nasal breathing mode can be adopted as the better breathing mode of the patients in nonanalgesic and sedative gastroscopy, which can reduce the adverse reactions related to the examination and, at the same time, improve the tolerance and comfort of the patients during the examination. In addition, to ensure smooth operation of the examination, endoscopists should continuously improve the proficiency and gentle operation of endoscopy. Nasal breathing is simple and easy for the patient and can effectively avoid the occurrence of anesthesia-related adverse reactions during gastroscopy with sedation and analgesia. This method has no additional cost, so the patients will not have economic pressure and burden. Therefore this method is more worthy to be popularized in primary hospitals.

## Figures and Tables

**Figure 1:** Mode of nasal inhalation and exhalation.

**Figure 2:** Mode of nasal inhalation and oral exhalation.

**Figure 3:** Visual analog scale (VAS).

**Figure 4:** Comparison of the cumulative term of adverse reactions between the two groups: *P* < 0.01.

**Figure 5:** Comparison of VAS scores between the two groups: *P* < 0.01.

**Table 1:** Comparison of general conditions between the two groups.

Items	Groups		*T*	*P*
	A group	B group		
Age	50.5 ± 12.52	51.23 ± 10.26	0.25	0.805
BMI	24.05 ± 1.02	23.78 ± 0.95	0.38	0.709

**Table 2:** Comparison of changes in vital signs between the two groups before, during, and after gastroscopy ($\bar{x}\pm s$).

Items	Groups		*T*	*P*
	A group (*n* = 30)	B group (*n* = 30)		
MAP (mmHg)				
Before examination	102.77 ± 4.24	101.13 ± 4.82	0.50	0.620
During examination	122.28 ± 4.79	129.64 ± 7.03	−1.69	0.097
After examination	106.78 ± 3.66	107.1 ± 5.26	−0.10	0.923

HR (min)				
Before examination	78.37 ± 4.08	77.93 ± 4.74	0.14	0.893
During examination	109.87 ± 5.61	113.86 ± 5.83	−0.96	0.341
After examination	87.23 ± 4.4	87.9 ± 4.99	−0.19	0.847

SpO2 (%)				
Before examination	97.8 ± 0.45	97.7 ± 0.47	0.30	0.766
During examination	98.23 ± 0.56	97.69 ± 0.77	1.12	0.269
After examination	98.23 ± 0.4	98.21 ± 0.39	0.09	0.926

**Table 3:** Comparison of inspection completion rates between the two groups (case %).

Groups	Completion rates [case (%)]	
	Success	Failure
A group (*n* = 30)	30	0
B group (*n* = 30)	29	1
*χ * ^2^	1.017	
*P*	0.313	

The article "Clinical Observation of the Effect of Nasal Breathing on Nonanalgesic and Sedative Gastroscopy" was retracted in 2023. Reasons: signs of a paper mill; suspected computer-generated content; unreliable results or conclusions; concerns about the data.

**Table 4:** Comparison of the incidence of adverse reactions of gastroscopy between the two groups (case %).

Groups	Belching	Nausea	Cough	Throat discomfort	Restlessness	Chest tightness
A group (*n* = 30)	20 (0.67)	15 (0.50)	6 (0.20)	3 (0.10)	0 (0.00)	0 (0.00)
B group (*n* = 30)	24 (0.80)	23 (0.77)	9 (0.30)	5 (0.17)	2 (0.67)	1 (0.03)
*χ * ^2^	1.364	4.593	0.800	0.577	2.069	1.017
*P*	0.243	0.032	0.371	0.448	0.150	0.313

## Data Availability

The datasets generated during and/or analyzed during the current study are not publicly available due to the sensitivity and data use agreement.
